# Comparison of Different Risk Scores for Prediction of In-Hospital Mortality in STEMI Patients Treated with PPCI

**DOI:** 10.1155/2022/5389072

**Published:** 2022-12-30

**Authors:** Chih-Hwa Wang, Hui-Ting Wang, Kuan-Han Wu, Fu-Jen Cheng, Cheng-I. Cheng, Chia-Te Kung, Fu-Cheng Chen

**Affiliations:** ^1^Department of Emergency Medicine, Kaohsiung Chang Gung Memorial Hospital, Chang Gung University College of Medicine, Kaohsiung, Taiwan; ^2^Division of Cardiology, Department of Internal Medicine, Kaohsiung Chang Gung Memorial Hospital, Chang Gung University College of Medicine, Kaohsiung, Taiwan

## Abstract

**Background:**

Several risk scores have been developed to predict and analyze in-hospital mortality and short- and long-term outcomes of ST-elevation myocardial infarction (STEMI) patients after primary percutaneous coronary intervention (PPCI); these can classify patients as having a high or low risk of death or complications.

**Objective:**

To compare the prognostic precision of four risk scores for predicting in-hospital mortality in patients with STEMI treated with PPCI.

**Methods:**

We performed a retrospective cohort analysis of patients with STEMI who underwent PPCI between 2012 and 2019 (*N* = 1346). GRACE (Global Registry of Acute Cardiac Events), CADILLAC (Controlled Abciximab and Device Investigation to Lower Late Angioplasty Complications), Zwolle, and TIMI (Thrombolysis in Myocardial Infarction) risk scores were calculated for each patient according to different variables. We evaluated the predictive accuracy of these scores for in-hospital mortality using the *C* statistic, which was obtained using logistic regression and receiver operating characteristic curves.

**Results:**

The GRACE, CADILLAC, Zwolle, and TIMI risk scores all had good predictive precision for in-hospital mortality, with C statistics ranging from 0.842 to 0.923. The GRACE and CADILLAC risk scores were found to be superior.

**Conclusions:**

All GRACE, CADILLAC, Zwolle, and TIMI risk scores showed a high predictive value for in-hospital mortality due to all causes in patients with STEMI treated with PPCI. The GRACE and CADILLAC risk scores revealed a better accuracy for predicting in-hospital mortality than the Zwolle and TIMI risk scores.

## 1. Introduction

Acute coronary syndrome (ACS) is a common disease seen in the emergency department (ED), and patients with ACS are classified as having ST-elevation myocardial infarction (STEMI), non-ST-elevation myocardial infarction (NSTEMI), and unstable angina according to electrocardiography (ECG) findings and cardiac marker enzyme levels. In patients with STEMI with total coronary occlusion, necrosis and death of the heart muscle can lead to lethal cardiac arrhythmias and even cardiac arrest. Therefore, it is crucial that patients with STEMI be started on reperfusion therapy, including fibrinolytic therapy and primary percutaneous coronary intervention (PPCI), at the earliest. Despite recent improvements in medical care, morbidity and mortality rates of patients with STEMI remain high [1, 2]. In-hospital mortality after PPCI for STEMI patients ranges from 2.5% to 9.4% in Japan, from 2.2% to 6.1% in Europe, and from 5.7% to 6.3% in the United States [3–5].

Several risk scores have been developed to predict and analyze the in-hospital mortality of STEMI patients after PPCI, which can classify patients as having a high or low risk of death or complications [6–10]. The Thrombolysis in Myocardial Infarction (TIMI) risk score is a simple method that was initially derived from fibrinolytic-treated patients with STEMI to predict 30-day mortality. It was also found to be useful for predicting in-hospital mortality in STEMI patients treated with PPCI [7, 11]. The Global Registry of Acute Cardiac Events (GRACE) risk score is a widespread tool and was developed from a large population of patients with ACS and was used for predicting in-hospital mortality [8]. It was recommended by the European Society of Cardiology for risk stratification in patients with NSTEMI [12]. The Zwolle score was developed to predict 30-day mortality and identify low-risk STEMI patients who could be discharged early after PPCI [9]. The Controlled Abciximab and Device Investigation to Lower Late Angioplasty Complications (CADILLAC) risk score was developed to predict 30-day mortality and one-year mortality of STEMI and NSTEMI patients after PPCI [10, 13].

Several studies have compared the aforementioned risk scores to predict short-term and long-term outcomes in patients with STEMI treated with PPCI, but their conclusions are quite different [14–18]. Chen et al. reported that the GRACE risk score was more accurate in predicting long-term mortality (up to three years) in Asian patients with myocardial infarction, including STEMI and NSTEMI [19]. A study by Littnerova et al. concluded that GRACE appeared to be the most suitable tool for the prediction of outcomes over a longer follow-up period [16]. We are of the opinion that these risk scores were initially designed for estimating short-term mortality and are the most timely and important tools for the prediction of in-hospital mortality. The conclusions of these studies for the comparison of various scores are not consistent, possibly due to differences in race, diet, and living habits. We compared the GRACE, CADILLAC, Zwolle, and TIMI risk scores to predict in-hospital mortality in STEMI patients undergoing PPCI, to see if the results differed from previous studies, and to examine the reasons for the differences.

## 2. Methods

### 2.1. Study Design

This single-center retrospective study was conducted at the Kaohsiung Chang Gung Memorial Hospital, a medical center with more than 2500 inpatient beds and 5500 servants providing primary and tertiary referral care in Southern Taiwan. PPCI services have been available for 24 hours a day and 7 days a week since 2001, and over 150 STEMI patients are treated annually. The study period was from January 2012 to December 2019. All patient and physician data were deidentified, and the study protocol was approved by the Ethics Committee of Chang Gung Memorial Hospital (Approval number: 202000548B0). Owing to the retrospective nature of the study, a waiver of informed consent was granted.

### 2.2. Study Setting and Participants

We enrolled patients with STEMI who presented to the ED during the study period. These patients had developed symptoms within 12 h prior to presenting themselves in the ED and subsequently underwent PPCI. The exclusion criteria included patients presenting to the ED with out-of-hospital cardiac arrest and patients whose collected data were insufficient. The patients we included were all of the Asian ethnicity.

### 2.3. Measurement and Data Collection

The risk scores mentioned above are influenced by multiple factors, including baseline condition and underlying disease; age, weight, creatinine/renal insufficiency, diabetes mellitus (DM), hypertension, and angina pectoris; ischemic condition on admission—blood pressure, heart rate, anterior myocardial infarction or left bundle branch block (LBBB), Killip class (evaluation of patient's severity in the prediction of patient's mortality risks according to the physical examination and degree of heart failure) [20], and ischemia time; post-PPCI condition; TIMI-3 flow grade assessment after PPCI (grade 3 indicating normal blood flow in the coronary artery after thrombolysis) [21], and left ventricular ejection fraction (LVEF) calculated by transthoracic echocardiography. We retrospectively evaluated all these factors and added time intervals consisting of symptom-to-balloon, door-to-ECG, and door-to-balloon times. Laboratory data and vital signs were recorded at the presentation. The underlying diseases of the patients were based on their statements and previous medical records.

### 2.4. Risk Scores and Factors

The GRACE risk score consisted of age, systolic blood pressure, heart rate, Killip class, elevated cardiac enzyme levels, and serum creatinine levels. The CADILLAC risk score included age, TIMI flow after PPCI, triple-vessel disease, LVEF, Killip class, renal insufficiency (estimated creatinine clearance <60 mL/min), and anemia (hematocrit <39% in men and <36% in women). The Zwolle risk score included age, Killip class, anterior infarction, ischemia time, TIMI flow after PPCI, and triple-vessel disease. The TIMI risk score included age, systolic blood pressure, heart rate, Killip class, weight, DM, hypertension, angina pectoris, anterior wall MI or LBBB, and duration of ischemia.

### 2.5. Endpoint

The endpoint of this study was in-hospital mortality due to all causes in STEMI patients who underwent PPCI after admission.

### 2.6. Statistical Analysis

Continuous variables were presented as mean ± standard deviation (SD) or median with interquartile range and were analyzed using Student's *t*-test or the Mann–Whitney *U* test. Categorical variables were presented as numbers and percentages and were compared using the chi-squared (*χ*^2^) test or Fisher's exact test. The discriminative potential of the risk scores was determined using the area under the receiver operating characteristic curve (AUROC) to describe the diagnostic precision of the risk scores [22]. The optimal cutoff thresholds were resolved using the Youden index. Statistical significance was set at *p* < 0.05. The AUROC for these scores was compared using the DeLong test. All analyses were performed using IBM SPSS Statistics for Windows, version 25 (IBM Corp., Armonk, NY, USA), and the receiver operating characteristic (ROC) curves for clinical event models were compared using MedCalc® Statistical Software version 19.7.2 (MedCalc Software Ltd., Ostend, Belgium; https://www.medcalc.org; 2021).

## 3. Results

### 3.1. Study Group

A total of 1,436 STEMI patients underwent PPCI between 2012 and 2019. This study included 1,346 patients after excluding those with out-of-hospital cardiac arrest (*n* = 21) and insufficient data collection (*n* = 69). In total, 1,274 patients survived and were discharged, while 72 died while admitted to the hospital. The in-hospital mortality rate was 5.3%.

### 3.2. Statistical Analysis of Other Affecting Factors

The baseline characteristics, vital signs, and laboratory data of survivors and nonsurvivors are listed in Table 1. Nonsurvivors were older (68.3 ± 13.4 years compared to 60.1 ± 12.5 years in survivors), and there were more women (33.3% compared to 14.8% in survivors). Nonsurvivors had a lower systolic blood pressure (115 ± 40 mmHg compared to 140 ± 34 mmHg in survivors), higher heart rate (92 ± 30 bpm compared to 79 ± 21 bpm in survivors), lower hemoglobin (12.9 g/dL compared to 14.6 g/dL in survivors), lower hematocrit (38.7% compared to 43.1% in survivors), higher blood sugar (239 mg/dL compared to 157 mg/dL in survivors), higher creatinine (1.6 mg/dL compared to 1.1 mg/dL in survivors), higher AST (73 U/L compared to 32 U/L in survivors), and higher troponin-I (0.81 ng/mL compared to 0.12 ng/mL in survivors) levels, and there were more nonsurvivors with Killip class II-IV (88.9% compared to 35.6% in survivors). Angiographic features, results, and clinical outcomes are listed in Table 2. Additionally, we found that nonsurvivors had a longer symptom-to-balloon time (4.1 hours compared to 3.1 hours in survivors); there were fewer nonsurvivors with postprocedural TIMI-3 flow (84.7% compared to 94.8% in survivors) and more with multivessel disease (88.9% compared to 64.3% in survivors). The nonsurvivors had longer lengths of hospital stay (10.6 days compared to 4.8 days in survivors) and a lower LVEF (39% compared to 55% in survivors).

### 3.3. Characteristic Curve Analysis of the Risk Scores

The risk scores calculated by GRACE, CADILLAC, Zwolle, and TIMI are shown in Table 3, and they all scored higher in nonsurvivors. The median GRACE risk scores were 234 for nonsurvivors and 139 for survivors, respectively. The median CADILLAC risk score was 12 for nonsurvivors and three for survivors. The median Zwolle risk score was 12 for nonsurvivors and three for survivors. The median TIMI risk scores were seven for nonsurvivors and four for survivors. The ROC curves of the four risk scores for predicting in-hospital mortality are shown in Figure 1. AUROC was calculated, and the results were as follows: GRACE (0.918; 95% CI, 0.902–0.932), CADILLAC (0.888; 95% CI, 0.870–0.905), Zwolle (0.854; 95% CI, 0.834–0.873), and TIMI (0.822; 95% CI, 0.800–0.842). Youden's indices of GRACE, CADILLAC, Zwolle, and TIMI were 0.7154, 0.6414, 0.6042, and 0.5269, respectively, as shown in Table 4.

Among patients with STEMI who underwent PPCI, mortality was higher in women than in men, particularly in younger women [23–25]. Furthermore, delays in door-to-balloon and symptom-to-door times were associated with increased mortality [26, 27]. Therefore, we include age, sex, and symptom-to-balloon time as adjustment factors in the regression analysis. The ROC curves adjusted for age, sex, and symptom-to-balloon time are shown in Figure 2. AUROC was calculated, and the results were as follows: GRACE (0.923; 95% CI, 0.907–0.937), CADILLAC (0.895; 95% CI, 0.877–0.911), Zwolle (0.878; 95% CI, 0.859–0.895), and TIMI (0.842; 95% CI, 0.822–0.861). Whether AUROC was unadjusted or adjusted for the four risk scores, the GRACE risk score demonstrated the best discriminative precision in the prediction of in-hospital mortality in patients with STEMI treated with PPCI. The results of the DeLong test to compare the unadjusted and adjusted AUROC of each score are shown in Table 5. No difference was observed between GRACE and CADILLAC for adjusted AUROC of each risk score. Nevertheless, the GRACE risk score showed a statistically superior trend compared with the Zwolle and TIMI risk scores alone.

## 4. Discussion

We compared the GRACE, CADILLAC, Zwolle, and TIMI risk scores to predict in-hospital mortality in patients with STEMI treated with PPCI and found that the four risk scores exhibited a good level of prediction of in-hospital mortality. Furthermore, the GRACE and CADILLAC risk scores demonstrated better accuracy than the other two risk scores.

Most studies have concluded that the predictive power of the GRACE risk score is excellent [16–19]. However, Lev et al. indicated that the GRACE risk score had poor quality in the prediction of 30 days mortality in patients with STEMI treated with PPCI, and the *C* statistic of the GRACE risk score was 0.471 [14]. Our results differ from those of their study because they excluded patients with cardiogenic shock or cardiac arrest, which accounted for a significant portion of the GRACE risk score weighting. Our study did not exclude patients with cardiogenic shock. The exclusion of these patients in other studies may have contributed to the poor predictive value of the GRACE score for evaluating the STEMI population in those studies.

The predictive power of the TIMI risk score was slightly inferior in our patients compared with the other risk scores. The patients in the study group related to the TIMI risk scores or even the original study of the TIMI score were mostly of European and American ethnicity. However, the patients in our study group were all of the Asian ethnicity. There are many differences between races, many of which contribute to the cardiovascular risk. Factors such as genetics (different waist-to-hip ratios and obesity trends), dietary habits (fast food, wheat, and rice products), and lifestyle (physical activity, smoking prevalence, and low or high alcohol intake) play a role [28–30]. This also leads to different weight standards among races. However, the TIMI risk score uses body weight as an indicator, which may have affected the performance of the TIMI risk score in our study. According to a study conducted by the Korean Acute Myocardial Infarction Registry (KAMIR), body mass index (BMI) is positively correlated with 6 months of mortality in patients with STEMI [31]. We recommend converting patients' weight to BMI to improve the accuracy of the TIMI score to correct for differences between races.

The studies by Mendez-Eirn et al. and Littnerova et al. pointed out that the GRACE and CADILLAC risk scores had a better prediction of 30-day mortality in patients with STEMI receiving PPCI [15, 16]. These results are similar to those in our study. The GRACE risk score includes eight variables with a fairly complex scoring system for age, heart rate, systolic blood pressure, and creatinine level, with different scores established for these continuous variables. It also highlights variables associated with clinical presentation (Killip class and cardiac arrest on admission). Although ECG ST-segment deviation and elevated myocardial injury markers on admission were relatively unimportant in patients with STEMI, they did not affect the excellent predictive power of the GRACE risk score. The GRACE risk score was superior to the Zwolle and TIMI risk scores, especially for early mortality. From a statistical perspective, the GRACE model provides more complete information for these variables.

Regarding the CADILLAC risk score, it had a unique indicator different from the other risk scores, which was “anemia.” It has become a strong predictor of mortality in patients with ACS. In an analysis of 422,855 patients with ACS, Mamas et al. concluded that anemia was independently associated with 30‐day (OR 1.28, 95% CI 1.22–1.35) and 1‐year mortality (OR 1.31, 95% CI 1.27–1.35) [32]. In addition, a common variable for GRACE and CADILLAC risk scores was the serum creatinine level. A previous study by Anavekar et al. revealed that even mild renal disease is a major risk factor for cardiovascular complications in patients with myocardial infarction [33]. Several studies have also found that acute kidney injury or chronic renal failure is an independent predictor of in-hospital mortality in patients with STEMI complicated with cardiogenic shock [34–36]. These are the reasons why GRACE and CADILLAC scores show excellent accuracy in predicting in-hospital mortality in STEMI patients undergoing PPCI.

Although several studies have compared different risk scores to predict short-, mid-, and long-term mortality and outcomes in STEMI patients undergoing PPCI, these risk scores are not very accurate for long-term prediction [14–18]. In addition, these risk scores were not originally designed to predict long-term mortality. Therefore, we believe that it is important for clinicians to compare these risk scores to predict in-hospital mortality in patients with STEMI undergoing PPCI.

## 5. Limitations

Our study had some limitations. Firstly, the study group was a single medical center study with a small sample size and an ethnic Asian study group. However, our study can serve as a model for further studies comparing different risk models across different ethnic groups. Secondly, this study was limited by its retrospective nature. Although every effort has been made to use regression statistical controls, some confounding factors may not have been accounted for. Thirdly, we included all-cause in-hospital mortality rather than purely cardiac in-hospital mortality. Although some patients may die from sepsis or other diseases unrelated to cardiac causes, we believe that myocardial infarction may indirectly affect medical conditions, leading to noncardiac mortality.

## 6. Conclusions

All GRACE, CADILLAC, Zwolle, and TIMI risk scores showed a high predictive value for all-cause in-hospital mortality in patients with ST-elevation myocardial infarction treated with PPCI. However, the GRACE and CADILLAC risk scores revealed a better accuracy for predicting in-hospital mortality in patients with STEMI treated with PPCI compared to the Zwolle and TIMI risk scores.

## Figures and Tables

**Figure 1:** Receiver operating characteristic curves of scoring models for in-hospital mortality.

**Figure 2:** Receiver operating characteristic curves of scoring models for in-hospital mortality adjusted by age, sex, creatinine, and symptom-to-balloon time.

**Table 1:** Baseline characteristics, vital signs, and laboratory data.

Variables	All patients (*n* = 1346)	Survivor (*n* = 1274)	Nonsurvivors (*n* = 72)	*P* value
Age (years)	60.5 ± 12.7	60.1 ± 12.5	68.3 ± 13.4	<0.001^*∗*^
Male gender	1134 (84.2)	1086 (85.2)	48 (66.7)	<0.001^*∗*^
Body mass index (kg/m^2^)	25.7 ± 4.0	25.7 ± 3.9	26.2 ± 4.8	0.371
Diabetes mellitus	535 (39.7)	493 (38.7)	42 (58.3)	0.001^*∗*^
Hypertension	889 (66.0)	842 (66.1)	47 (65.3)	0.899
Dyslipidemia	1034 (76.8)	983 (77.2)	51 (70.8)	0.250
Current smoking	760 (56.5)	730 (57.3)	30 (41.7)	0.01^*∗*^
Previous myocardial infarction	119 (8.8)	107 (8.4)	12 (16.7)	0.029^*∗*^
Systolic blood pressure^a^	138 ± 35	140 ± 34	115 ± 40	<0.001^*∗*^
Heart rate^a^	80 ± 21	79 ± 21	92 ± 30	<0.001^*∗*^
Anterior ST elevation	694 (51.6)	660 (51.8)	34 (47.2)	0.469
White blood cell count (k/mm^3^)^a^	10.9 (8.8–13.7)	10.8 (8.7–13.6)	12.0 (10.2–14.5)	0.042^*∗*^
Hemoglobin (g/dL)^a^	14.5 (13.2–15.6)	14.6 (13.3–15.7)	12.9 (10.8–14.5)	<0.001^*∗*^
Hematocrit (%)	42.9 (39.4–45.9)	43.1 (39.6–46.0)	38.7 (33.0–42.8))	<0.001^*∗*^
Platelet count (k/mm^3^)^a^	219 (184–259)	219 (185–259)	216 (176–275)	0.746
Sugar (mg/dL)^a^	159 (131–221)	157 (130–215)	239 (161–348)	<0.001^*∗*^
Creatinine (mg/dL)^a^	1.1 (0.9–1.4)	1.1 (0.9–1.3)	1.6 (1.2–2.8)	<0.001^*∗*^
AST (U/L)^a^	33 (25–51)	32 (25–48)	73 (41–211)	<0.001^*∗*^
Troponin-I (ng/mL)^a^	0.13 (0.03–0.90)	0.12 (0.03–0.79)	0.81 (0.16–9.82)	<0.001^*∗*^
Killip class II-IV^a^	517 (38.4)	453 (35.6)	64 (88.9)	<0.001^*∗*^

Data are expressed as mean ± SD or *n* (%) or median (25th—75th percentile). ^a^: All the data were measured upon presentation. ^*∗*^*P* < 0.05.

**Table 2:** Angiographic features, results, and clinical outcomes.

Variables	All patients (*n* = 1346)	Survivor (*n* = 1274)	Nonsurvivors (*n* = 72)	*P* value
Symptom-to-balloon time (hours)	3.1 (2.1–4.9)	3.1 (2.1–4.8)	4.1 (2.8–6.6)	0.001^*∗*^
Symptom-to-door time (hours)	2.1 (1.1–3.8)	2.1 (1.1–3.8)	2.9 (1.3–4.9)	0.039^*∗*^
Door-to-ECG time (minutes)	4 (2–6)	4 (2–6)	5 (3–8)	0.097
Door-to-cath room time (minutes)	33 (25–45)	33 (24–44)	47 (35–64)	<0.001^*∗*^
Reperfusion time (minutes)	17 (14–22)	17 (14–21)	23 (17–30)	<0.001^*∗*^
Door-to-balloon time (minutes)	52 (43–66)	52 (42–64)	72 (55–94)	<0.001^*∗*^
Postprocedural TIMI-3 flow	1269 (94.3)	1208 (94.8)	61 (84.7)	0.002^*∗*^
Stenting	1302 (96.7)	1232 (96.7)	70 (97.2)	1.000
Multivessel disease (≥2 vessels)	883 (65.6)	819 (64.3)	64 (88.9)	<0.001^*∗*^
Length of hospital stay (days)	4.9 (3.6–7.2)	4.8 (3.6–7.0)	10.6 (4.7–17.0)	<0.001^*∗*^
LVEF	55 (46–65)	55 (47–65)	39 (29–52)	<0.001^*∗*^
In-hospital mortality	72 (5)	—	—	—

Data are expressed as mean ± SD or *n* (%) or median (25^th^–75^th^ percentile). ECG: electrocardiography; LVEF: left ventricular ejection fraction; TIMI: thrombolysis in myocardial infarction. ^*∗*^*P* < 0.05.

**Table 3:** Risk scores.

Scores	All patients (*n* = 1346)	Survivor (*n* = 1274)	Nonsurvivors (*n* = 72)	*P* value
GRACE	141 (117–179)	139 (115–172)	234 (210–260)	<0.001^*∗*^
CADILLAC	4 (2–7)	3 (0–7)	12 (8–14)	<0.001^*∗*^
ZWOLLE	4 (2–8)	3 (2–7)	12 (10–13)	<0.001^*∗*^
TIMI	4 (2–6)	4 (2–6)	7 (6–10)	<0.001^*∗*^

Data are expressed as median (25^th^—75^th^ percentile) ^*∗*^*P* < 0.05.

**Table 4:** The AUROC, adjusted AUROC, sensitivity, specificity, Youden's index, and cut-off point of each risk score.

Scores	AUROC	95% CI	Adjusted AUROC^*∗*^	95% CI	Sensitivity	Specificity	Youden's index	Cut-offpoint
GRACE	0.918	0.902–0.932	0.923	0.907–0.937	0.8472	0.8681	0.7154	197
CADILLAC	0.888	0.870–0.905	0.895	0.877–0.911	0.9028	0.7386	0.6414	6
ZWOLLE	0.854	0.834–0.873	0.878	0.859–0.895	0.8750	0.7292	0.6042	6
TIMI	0.822	0.800–0.842	0.842	0.822–0.861	0.8056	0.7214	0.5269	5

^*∗*^Adjusted by age, sex, creatinine, and symptom-to-balloon time.

**Table 5:** Comparison of AUROC of the GRACE, CADILLAC, Zwolle, and TIMI.

Comparison	Unadjusted AUROC		Adjusted AUROC	
	*Z*	*P* value	*z*	*P* value
GRACE vs CADILLAC	1.775	0.0759	1.734	0.0830
GRACE vs ZWOLLE	4.275	<0.0001^*∗*^	3.836	0.0001^*∗*^
GRACE vs TIMI	5.907	<0.0001^*∗*^	4.958	<0.0001^*∗*^
CADILLAC vs ZWOLLE	1.694	0.0903	1.017	0.3093
CADILLAC vs TIMI	3.234	0.0012^*∗*^	3.836	0.0071^*∗*^
ZWOLLE vs TIMI	1.605	0.1084	2.301	0.0214^*∗*^

^*∗*^ *P* < 0.05.

## Data Availability

The data that support the findings of this study are available on request from the corresponding author.
